# Analysis of Coupling Coordination Degree between Big Health Industry and Pension Service

**DOI:** 10.1155/2022/6427024

**Published:** 2022-03-12

**Authors:** Liqiong Luo

**Affiliations:** School of Management, Wuhan College, Wuhan 430212, Hubei, China

## Abstract

With the aging of the population, the problem of providing for the aged has been paid more and more attention. The big health industry and old-age care services will complement and promote each other in terms of industrial factors, industrial layout, and policy linkage and form a coupling effect in this process. Hospital services and pension services are professional property service formats, and they are also the exploration achievements of the property management industry in implementing the supply-side structural reform, transformation, upgrading, and development and are indispensable forces for the property management industry to participate in building a better life. The health and happiness of the elderly is an important symbol of social civilization and progress, and it is also an important content of implementing the Healthy China Action. The pension industry serving the healthy life of the aged population will form a huge demand for the big health industry, and its development will drive the big health industry. Based on the background of the big health system, this paper analyzes the current situation and crux of the development of aged care services in China and puts forward ways to improve the quality of aged care services by optimizing the effective supply of aged care services, improving the environment of aged care services, and strengthening the precise supervision of aged care services.

## 1. Introduction

With the continuous improvement of people's living standards, health has become a hot topic. Promoting the integration and development of preventive health care, medical services, health care, and other health service industries and building a “great health” service system covering the whole life cycle of residents from gestation to pension are in line with the new normal of economic and social development and the new situation of health and family planning reform and development [1, 2]. The great health industry is involved in many fields of production, management, and service, such as medical treatment, medicine, health preservation, health care, and pension industry [3]. In the field of social economy, the coupling research is mainly applied to the relationship between various industries, economy, and environment and has more mature results [4]. With the central government's vigorous advocacy of “building a healthy leisure and health-keeping capital in China,” China takes the big health industry as the center, expands the health care service economy as the radius, and implements universal promotion in urban economy and quality of life to promote the comprehensive and harmonious development of the health industry [5]. The great health industry focusing on medical treatment, life sciences, hygiene, and health care, as a whole industrial chain covering health service, health production, and health management is stepping into the road of rapid development [6]. Hospital services and old-age care services are professional property service formats, and they are also the exploration achievements of the property management industry in implementing the supply-side structural reform, transformation, upgrading, and development and are an indispensable and important force for the property management industry to participate in building a better life [7]. The health and happiness of the elderly is an important symbol of social civilization and progress, and it is also an important content of implementing the Healthy China Action [8].

With the country putting forward a series of policies on health service and pension industry, China's big health industry has also ushered in a golden period of development [8]. It is a natural law that the physical function of the elderly deteriorates and their health condition declines, and medical and health services are an objective necessity to maintain the quality of life of the elderly [9]. Healthy living is the foundation of the aged population's life or providing for the aged. The development of the big health industry can bring better health care products and services and more scientific health care management and provide better technical support and health services for the development of health-care-based pension industry [10]. Under the broad vision of reform and opening up, the combination of medical care and nursing care is the supply-side problem in the construction of the old-age service industry system, which should be promoted with reform ideas, open concepts, and innovative thinking [11]. The development of the pension industry will also provide a platform for the development of the big health industry. The pension industry that serves the healthy life of the elderly population will form a huge demand for the big health industry, and its development will drive the big health industry [12]. The health and happiness of the elderly is an important symbol of social civilization and progress, and it is also an important content of implementing the Healthy China Action. As a major livelihood issue, the old-age pension has gradually attracted the attention of the state and the public [13]. With the vigorous development of the big health industry, the project operation has gradually stabilized. If it can attract a large number of stable and high-quality user groups, its market potential will be unpredictable [14].

The big health industry and old-age care services will complement and promote each other in terms of industrial factors, industrial layout, and policy linkage and form a coupling effect in this process. With the aging of the population, the problem of providing for the aged has attracted more and more attention [15]. As a new industry, the old-age care industry, especially serving the elderly, is in the ascendant, including old-age recuperation, old-age supplies, old-age services, old-age real estate, old-age culture, old-age travel, old-age catering, and so on [16]. As a global concept, Great Health focuses on people's food, clothing, housing, life, and death and pursues full-course, comprehensive, and all-factor health care, thus realizing individual physical and mental health. Pension is not only an industrial problem but also a social problem and a responsibility problem [17]. In China, there is still much room for progress and improvement in the industrial structure, operational capability, and industrial transformation of the big health care industry in its initial stage [18]. We must focus on making the old-age care industry flexible, market-oriented, and diversified; integrating deep-rooted traditional formats with emerging formats; providing different types of healthy old-age care products; and creating a new road of great healthy old-age care services in line with socialism with Chinese characteristics [19]. Based on the background of the big health system, this paper analyzes the current situation and crux of the development of aged care services in China and puts forward ways to improve the quality of aged care services by optimizing the effective supply of aged care services, improving the environment of aged care services, and strengthening the precise supervision of aged care services.

## 2. The Crux of the Reform of Pension Service in China

The acceleration of population aging will increase the pressure on social security and public services, weaken the demographic dividend, and continuously affect social vitality, innovation power, and potential economic growth rate, which is an important risk and challenge for population development in the new era. In the field of aged care services, the big health system, with the help of big data technology, explores and integrates the health big data resources of the elderly and breaks the boundaries between medical treatment, rehabilitation, maintenance, and old-age care by implementing full-course, comprehensive, and all-factor care, thus improving the quality of aged care services and pursuing the physical health of the elderly while realizing their mental health and mental health [20]. The combination of medical care and nursing focuses on the community and the family. The most important thing of medical and nursing services is to shift the center of gravity of medical and health resources and extend basic medical and health services and services for the elderly to communities and families. Nowadays, the state vigorously supports the old-age service industry in the big health industry. The most striking and typical one is the preferential policies for the old-age service, which makes the capital market and entrepreneurs see opportunities and hopes. Under the guidance of scientific and technological innovation, the content, format, and system of aged care services are constantly enriched. On the other hand, the development of old-age service mainly provides market elements for the development of big health industry, and the old-age service groups are gradually covered by young and energetic old people, with diversified development of old-age models such as ecological old-age care, intelligent old-age care, and residential old-age care.

With the acceleration of population aging and the increasing number of elderly people in China, there is an urgent need to reform the old-age service. By integrating the concept of great health, a model of old-age service in line with China's national conditions is established. However, at present, China's old-age care system still needs to be improved to meet the realistic demands of social old-age care by improving the quality of old-age care services. The old-age service provides a new development idea for the big health industry, which enriches the service content of the old-age service. The integration of resources required by the model of combining medical care with old-age care is not a simple addition of two kinds of resources, but specialized medical resources should be supplied to the old-age care field in a hierarchical and diversified way. Medical and health institutions are recognized and managed by the health department, and medical insurance reimbursement is managed by the social security department [21]. Combining medical care with nursing care, we should constantly improve the socialization system of old-age service; pay attention to hardware, operation, and service in the streets; and realize the enhancement of modern hardware functions. On the one hand, based on the characteristics that pension service is different from family pension and institutional pension, under the background that family pension function is weakening day by day, facing the huge demand for pension service for the elderly, the elderly health service industry came into being [22]. On the other hand, the health care industry in the big health industry promotes the combination of medical care and nursing care, and the innovation of smart pension and healthy pension real estate brought by scientific and technological progress, and various pension communities broaden the connotation of pension service mode. The traditional community home-based aged care service model emphasizes life care and mainly provides services such as helping the elderly with meals and cleaning. It is out of touch with the current needs of the elderly, cannot meet all-round health care under the big health system, and cannot provide aged care services such as life care, culture and entertainment, medical care, spiritual comfort, and emergency assistance for the elderly.

## 3. Coupling and Coordination of Big Health Industry and Pension Service

### 3.1. Optimizing the Effective Supply of Pension Services in an All-Round Way

Under the big health system, China's old-age service reform must focus on the overall situation and meet diversified, convenient, and personalized service demands by constructing an all-round, multilevel, and three-dimensional old-age service system, including optimizing the supply of old-age services on the demand side, perfecting the old-age service environment, and supervising the quality of old-age services. With the country putting forward a series of policies on health service and pension industry, China's big health industry has also ushered in a golden period of development. It can be predicted that the big health industry will become the growth point of China's economic development, and China's old-age health service industry will also get a good opportunity for development [23]. In view of the combination of medical care and health care service system construction, it is necessary to clarify the rational management of the lead department, coordinate the innovation of management mechanism, and improve the smooth implementation of the policy guarantee measures for the combination of medical care and health care. The urban old-age service institution combining medical care with nursing care is the support and carrier of medical care with nursing care and is the key to promoting the development of the old-age care system combining medical care with nursing care. How to provide better quality and more valuable protection and services for the health care industry is a common problem faced by property owners. It has become the common value goal and pursuit of colleges, aged service enterprises, and the government to train high-quality aged service professionals needed by the development of aged service enterprises and the aged care for the elderly.

To optimize the effective supply of aged care services, we must start with improving the quality and efficiency of institutional aged care services. For example, we should actively improve China's pension service system and realize the diversified development of community pension, home pension, and institutional pension. In addition, with the increasingly severe aging situation of the population, the care of the elderly, disabled, and demented people has become an unavoidable problem in society. The care for this kind of elderly group has also shifted from basic old-age service needs to medical rehabilitation, culture and entertainment, and so on. For example, Table 1 shows the elderly's choice of pension methods in a survey of 200 elderly people over 60 years old who are not living in pension institutions.

Property service enterprises are located at the nodes of society and community, which are closest to the resources and users of the community, understand and are closer to the various needs of the community, and have the highest correlation with community grassroots organizations, various professional service departments, surrounding business circles, and service industries. Therefore, property service enterprises that serve community users for a long time have inherent advantages in providing “community home care for the aged.” From the perspective of the supply side of old-age services, social forces should be encouraged and supported to set up medical and nursing services and set up medical and nursing services and professional medical institutions such as rehabilitation and nursing for the elderly through the market-oriented operation. The pension service industry is a kind of public welfare industry, which is quite different from the traditional home-based pension model. Urban old-age service system should play a decisive role in the allocation of urban old-age service resources combined with medical care, mobilize the enthusiasm and creativity of social forces, expand the scope of basic old-age insurance, and comprehensively improve the service quality of old-age institutions, thus promoting the development of urban old-age service combined with medical care [24]. Most of the professional and technical talents in aged service enterprises are concentrated in mature fields such as medical services and financial services, while the gap of professional and technical talents in aged care services and some fields to be developed is large, which is far from meeting the market demand. After all, old-age services are different from other services, so the state cannot push all old-age services to enterprises and markets. The for-profit and public welfare of the aged service industry are not contradictory to each other but promote each other and play a role in the aged service together. We should encourage the rational transformation of medical resources and old-age resources, improve the service level of old-age services in medical institutions, and set up good medical institutions and medical and health management systems.

A survey of 399 elderly people living in old-age care institutions shows that the elderly who are willing to go to old-age care institutions account for the highest proportion of the total number of elderly people surveyed, as shown in Table 2.

The so-called great health actually refers to the implementation of “whole-course, comprehensive and all-factor care” around people's daily life, food, clothing, housing, transportation, birth, death, and illness, which pursues not only personality and physical health but also psychological and spiritual health. At the same time, the big health industry is also a green sunrise industry without borders. It can be perfectly integrated with the primary, secondary, and tertiary industries. At present, many grassroots medical and health service institutions have limited conditions and cannot ensure houses and venues that meet the requirements. In the process of the development of the aged service industry, the government's responsibility is to do a good job in top-level design, formulate policies and systems, and strengthen supervision, so as not to interfere too much with the behavior of enterprises. Governments at all levels should establish a scientific and predictable concept of medical care combined with the old-age service guarantee, strengthen the innovation of policy support system and mechanism, and incorporate the construction of medical care combined with old-age service system into the local economic and social development plan [25]. Building a team of high-quality and professional aged care service talents is the foundation of supporting the aged care service industry. At present, the shortage and mobility of aged care service talents have become the shortcomings of industry development. The aged service enterprises can share their worries for the government, and their vigorous development is the foundation for the healthy development of the aged service specialty. At the same time, their development and growth also need the guidance and assistance of the government. The collaborative training system of aged service talents in colleges and universities and aged service enterprises should be developed on the basis of relevant government policies and constantly innovated and adjusted according to the actual situation.

### 3.2. Improving the Elderly Service Environment

Under the big health system, the goal of China's pension service reform is to meet the needs of the elderly for all-round, multilevel, differentiated, and high-quality pension services. Therefore, to improve the old-age market system, we must create a good old-age service environment from the supply side. In addition, we should speed up the process of the credit system construction of service subjects in the aged care market and improve the transparency of service information of aged care institutions by carrying out service quality ratings of aged care enterprises and individuals, so as to improve the supervision ability and service level of the aged care service market and further optimize its business environment. To become bigger and stronger, enterprises need to find their own position. Property service enterprises should balance their mentality and seek more opportunities in the concept of win-win cooperation. Aging means a fundamental change in human structure, which will have a wide and far-reaching impact on economic, political, and social development. It is not related to social harmony and stability but also tests the wisdom of the government and society [26]. In the process of the development of the aged service industry, the investors who provide services for the aged population, whether they are enterprises or social organizations, should be able to obtain certain benefits. In form, take the road of diversity. Conditional old-age care institutions can apply for self-operated hospitals, clinics, and other specialized medical services and nursing institutions. It is also possible to establish diversified places for providing health services for the aged, such as health examination, health care, recuperation, and family community.

The motive force of cultivating aged service talents comes from external drive and internal drive. The external motive force comes from the demand of social development and policy drive, while the internal motive force comes from the expected benefit pursuit of all parties who need talents. Reliability reflects the stability or reliability of measurement tools, which is generally evaluated by the reliability coefficient, that is, the correlation coefficient of two measurement results is taken as the reliability coefficient. The overall coefficient of the elderly health evaluation index system is 0.65, which shows that the overall evaluation index system has high internal consistency. The dimensions and overall reliability coefficient of the health-related index field evaluation system are shown in Table 3.

In order to analyze the effects of fiscal and financial policies on the development of pension finance, a variable parameter state-space model is used to measure the dynamic effects of fiscal and financial policies on the development of pension finance. The regression model of variable parameter state-space model is expressed as follows:

(1) $$\begin{array}{c} y_{t}=\beta_{t}x_{t}+\mu_{t},\;t=1,2,\Lambda ,T. \end{array}$$

Among them, *y*_*t*_ is the dependent variable, *x*_*t*_ is the 1 × *m* explanatory variable vector, *β* is the *m* × 1 unknown parameter vector to be estimated, and *μ*_*t*_ is the disturbance term. The parameters estimated by the commonly used regression models are fixed during the sample period and are generally estimated by measuring models such as ordinary least squares method and instrumental variable method, specifically

(2) $$\begin{array}{c} y_{t}=\beta_{t}x_{t}+z_{t}\gamma +u_{t},\;t=1,2\Lambda ,T. \end{array}$$

Among them, *β*_*t*_ is a variable parameter, which reflects the change in the influence of the variable on the dependent variable at that time. It is assumed that *β*_*t*_ can be described by AR(1) as follows:

(3) $$\begin{array}{c} \beta_{t}=\phi \beta_{t-1}+\xi_{t}. \end{array}$$

It is further extended to AR(*p*) model while assuming

(4) $$\begin{array}{c} {\left(\mu_{t},\xi_{t}\right)}^{\prime }∼N\left[\left[\begin{array}{c} 0\\ 0 \end{array}\right],\left[\begin{array}{cc} \sigma_{t}^{2} & g\\ g & Q \end{array}\right]\right],\;t=1,2\Lambda ,T. \end{array}$$

Among them, *μ*_*t*_ and *ξ*_*t*_ are not necessarily independent of each other, but they obey a normal distribution with a covariance matrix of Q and cov(*μ*_*t*_, *ξ*_*t*_)=*g*, a mean of 0 and a variance of *σ*^2^.

Urban old-age service system should play a decisive role in the allocation of urban old-age service resources combined with medical care, mobilize the enthusiasm and creativity of social forces, expand the scope of basic old-age insurance, and comprehensively improve the service quality of old-age institutions, so as to promote the development of urban old-age service combined with medical care. Today, with the development of the Internet, the elderly have become a vulnerable group in a certain sense due to the decline of relearning ability and recognition ability. Therefore, the key to improving the consumption environment of old-age services is to protect the old-age consumption rights and interests. Based on the characteristics that the elderly are keen on keeping in good health and their risk identification ability is weak, they can actively carry out health knowledge propaganda and antifraud public welfare activities for the elderly, so as to enhance their risk identification ability of pension fraud. The pension service industry is a kind of public welfare industry, which is quite different from the traditional home-based pension model. Today's old-age care model can provide more care, more professional care, rehabilitation care, and emotional care for the elderly. The two-way referral service mechanism between old-age care institutions and medical institutions has not yet been established, and resources cannot be shared. Once the elderly get sick, they have to travel between families, medical institutions, and old-age care institutions. There is no established existing model to follow and use in China, let alone a unified and successful scheme to implement, and the institutional mechanisms of other developed countries are not suitable for China's actual situation. Pension institutions can establish a medical and nursing partnership with local hospitals, and the cooperative hospitals can provide medical and health services for contracted pension institutions in a fixed-point and directional manner. They can also support various market players by purchasing services and equity cooperation and increase the supply of medical and nursing services and products. In the process of building a healthy old-age service system combining medical care with nursing care, it is necessary to promote the reform of old-age medical care, promote the integration and development of medical care and old-age service, and analyze it according to specific work. Neither party can bear the pressure of long-term care expenditure alone. Only by establishing a scientific financial burden mechanism can the aging industry run sustainably for a long time.

## 4. Conclusion

The big health system breaks the boundaries between traditional medical treatment, rehabilitation, maintenance, and old-age care and has important theoretical guiding significance for improving the quality of old-age care and ensuring the physical health, mental health, and mental health of the elderly. Aging means a fundamental change in human structure, which will have a wide and far-reaching impact on economic, political, and social development. It is not only related to social harmony and stability but also tests the wisdom of the government and society. The motive force of cultivating aged service talents comes from external drive and internal drive. The external motive force comes from the demand of social development and policy drive, while the internal motive force comes from the expected benefit pursuit of all parties who need talents. In the process of building a healthy old-age service system combining medical care with nursing care, it is necessary to promote the reform of old-age medical care, promote the integration and development of medical care and old-age service, and analyze it according to specific work. Neither party can bear the pressure of long-term care expenditure alone. Only by establishing a scientific financial burden mechanism can the aging industry run sustainably for a long time. Urban old-age service system should play a decisive role in the allocation of urban old-age service resources combined with medical care, mobilize the enthusiasm and creativity of social forces, expand the scope of basic old-age insurance, and comprehensively improve the service quality of old-age institutions, so as to promote the development of urban old-age service combined with medical care.

## Figures and Tables

**Table 1:** Elderly people's choice of old-age care methods.

Projects	Pension type					
	Home		Community		Institutions	
	Number of people	Proportion (%)	Number of people	Proportion (%)	Number of people	Proportion (%)
Data	108	54	19	9.5	73	36.5

**Table 2:** Elderly people choose to go to integrated medical and elderly care institutions.

Content	Health status of the elderly					
	Self-care		Partly self-care		No self-care	
	Number of people	Proportion (%)	Number of people	Proportion (%)	Number of people	Proportion (%)
Willing	164	66.4	30	46.2	65	74.7
Unwilling	45	18.2	10	15.4	19	21.8
Not clear	38	15.4	25	38.5	3	3.4

**Table 3:** Dimensions and overall reliability coefficients of the health-related finger field evaluation system.

Dimensions	Number of indicators
Activity ability	16
Somatic function	10
Emotional character	8
Memory function	6
Healthy behavior	8
Social adaptability	9

## Data Availability

The data used to support the findings of this study are included within the article.
